# Relationship between Serum TSH Level and Adverse Pregnancy Outcome in Advanced Maternal Age

This article has been retracted.

**DOI:** 10.1155/2022/2063049

**Published:** 2022-04-15

**Authors:** Xiufang Shao, Kunhai Ren, Haiyan Tang, Yingling Xiu, Mian Pan

**Affiliations:** ^1^Gynaecology and Obstetrics, Fujian Maternity and Child Health Hospital, Fuzhou 350000, China; ^2^Clinical Lab, Fujian Maternity and Child Health Hospital, Fuzhou 350000, China

## Abstract

The purpose of this paper is to explore the relationship between serum thyroid-stimulating hormone (TSH) levels and adverse pregnancy outcomes in advanced maternal age. A total of 97 elderly parturient women who were treated in our hospital from June 2020 to March 2021 are included in this study. According to the TSH level, the parturient women are divided into three groups, including A (<0.25 *μ*IU/ml), B (>4.00 *μ*IU/ml), and C (0.25–4.00 *μ*IU/ml) groups. The clinical data of all parturients are collected and sorted out. The serum levels of TSH, free triiodothyronine (FT3), and free thyroxine (FT4) are measured by chemiluminescence immunoassay. The levels of immunoglobulin (Ig) A, IgG, and IgM are determined by immunoturbidimetry. The incidence of adverse pregnancy outcomes is analyzed. The birth weight and Apgar score of newborns in the three groups are compared. The TSH level in group A is significantly lower than that in groups B and C, but the levels of FT3 and FT4 in group A are notably higher than those in groups B and C (*P* < 0.05). The levels of IgA, IgG, and IgM in group A are significantly higher than those in groups B and C (*P* < 0.05). The incidence of adverse pregnancy outcomes in group C is 2.38%, which is obviously lower than the 20.00% in group A and 17.14% in group B (*P* < 0.05). The birth weight and Apgar score of infants in group A and group B are significantly lower than those in group C (*P* < 0.05). TSH has a great influence on the pregnancy outcome in advanced maternal age, which should be paid more attention in clinic.

## 1. Introduction

Thyroid disease is a common complication in obstetrics, and its prevalence is only lower than that of gestational diabetes. Once thyroid disease occurs during pregnancy, it not only endangers the physical and mental health of the pregnant woman, but also directly affects the thyroid function and endangers the long-term cognition of the fetus [1,2]. Elderly parturient women usually refer to women over 34-year old who have a great risk of intrauterine growth retardation and premature delivery [3,4]. It is a common type of high-risk pregnancy.

Due to the increased levels of human chorionic gonadotropin in pregnant women and the needs of growth and development in the fetus, it is very easy to cause abnormal thyroid hormone levels and endanger the normal metabolism of pregnant women. Once elderly parturient women with thyroid hormone disorders, it can significantly increase the hidden health risks of the mother and the fetus [5,6]. Therefore, it is the key to master the relationship between thyroid hormone level and pregnancy outcome in elderly women. In particular, it is important to pay attention to the influence of serum thyroid-stimulating hormone (TSH) level on pregnancy outcome, in order to avoid the incidence of adverse pregnancy outcome and ensure the safety of mother and baby [4].

Therefore, the purpose of this study is to explore the relationship between serum TSH level and adverse pregnancy outcome in advanced maternal age.

The rest of this paper is organized as follows: Section 2 is subjects and methods, followed by the comparison of thyroid hormone indexes among the three groups in Section 3. Thyroid disease is discussed in Section 4.  Section 5 shows the conclusion and future research suggestions.

## 2. Subjects and Methods

### 2.1. Subjects

This study is approved by the ethics committee of our hospital. All subjects sign informed consent. A total of 97 elderly parturient women who were treated in our hospital from June 2020 to March 2021 are included in this study. According to the TSH level, the parturient women are divided into three groups, including A (<0.25 *μ*IU/ml), B (>4.00 *μ*IU/ml), and C (0.25–4.00 *μ*IU/ml) groups. The inclusion criteria were as follows: (1) pregnant women over 34 years old; (2) informed consent is obtained from the subjects and their families; (3) gestational age of women who are 28–36 weeks, singleton pregnancy; and (4) women with complete clinical data. The exclusion criteria were as follows: (1) women with multiple pregnancy; (2) women with diseases such as diabetes, hypertension, thyroid diseases, autoimmune diseases, and inherited metabolic diseases before pregnancy; (3) women with consciousness or hearing impairment; and (4) women with heart, brain, liver, and kidney dysfunction, mental illness, or infectious diseases [19–21].

### 2.2. Detection of Biochemical Indexes

The fasting venous blood (5 ml) of all parturients is collected in the morning and centrifuged (3000 r/min) for 10 min. The serum was collected. The serum levels of TSH, free triiodothyronine (FT3), and free thyroxine (FT4) are measured by the Centaur XP automatic Chemiluminescence immunoassay system (Sinopharm Medical Supply Chain Service Company, Fuzhou, China) with the original kits according to the instructions. The levels of immunoglobulin (Ig) A, IgG, and IgM are determined using Siemens BNP II specific protein analyzer (Sinopagic Medical Supply Chain Service Co., Ltd., Fuzhou, China) and the original kit according to the manufacturer's protocol, using immunoturbidimetry.

### 2.3. Observation Indexes

The clinical data of all parturients are collected and sorted out. Serum levels of TSH, FT3, FT4, IgA, IgG, and IgM are collected. All pregnant women are followed up until delivery. The incidence of adverse pregnancy outcomes is collected. The birth weight and Apgar scores of newborns in the three groups are collected. The scoring standard of the Apgar score is as follows: 0–3 points for severe asphyxia; 4–7 points for mild asphyxia; and 8–10 points for normal.

### 2.4. Statistical Analysis

Statistical analysis is made by software SPSS17.0 (International Business Machines, Corp., Armonk, NY, USA). The measurement data are expressed as the mean± standard deviation (SD) and compared by the *t*-test. The counting data are expressed as percentage and compared by the *χ*^*2*^ test. Differences are considered statistically significant when *P* < 0.05.

## 3. Experimental Results and Analysis

There are 20 women in group A, 35 women in group B, and 42 women in group C. There are 12 primipara and 8 multiparas in group A. The average age of pregnant women in group A is 38.25 ± 1.02 years old, and the average gestational age is 31.45 ± 0.87 weeks. There are 19 primipara and 16 multiparas in group B. The average age of pregnant women in group B is 38.40 ± 1.11 years old, and the average gestational age is 31.60 ± 0.91 weeks. There are 24 primipara and 18 multiparas in group C. The average age of pregnant women in group C is 38.73 ± 1.16 years old, and the average gestational age is 31.87 ± 0.75 weeks. There is no difference in basic information among the three groups (*P* > 0.05).

### 3.1. Comparison of Thyroid Hormone Indexes among the Three Groups

As shown in Table 1, the TSH level in group A is significantly lower than that in group B and group C (*P* < 0.05). However, the levels of FT3 and FT4 in group A are notably higher in comparison with group B and group C (*P* < 0.05).

### 3.2. Comparison of Immune Indexes among the Three Groups

As shown in Table 2, the IgA level in group A is significantly higher than that in group B and group C (*P* < 0.01). Similarly, the IgG level in group A is notably higher in comparison with group B and group C (*P* < 0.05). Moreover, the IgM level in group A is obviously higher in comparison with group B and group C (*P* < 0.05).

### 3.3. Comparison of Adverse Pregnancy Outcomes among the Three Groups

As shown in Table 3, the pregnancy outcomes mainly included cesarean section, premature birth, birth defects, and healthy term infants. As shown in Table 3, the incidence of adverse pregnancy outcomes in group C is 2.38%, which is obviously lower than 20.00% in group A and 17.14% in group B (*P* < 0.05).

### 3.4. Comparison of Neonatal Status among Three Groups

As shown in Table 4, the birth weight of infants in group A and group B is significantly lower than those in group C (*P* < 0.05). Moreover, the Apgar scores of infants in group A and group B are notably lower than those in group C (*P* < 0.05).

## 4. Discussion

As a common clinical endocrine disease, thyroid disease is also a common multiple disease in pregnant women. It can directly affect fetal thyroid function and endanger long-term cognition, normal growth and development. In recent years, with the continuous changes in domestic fertility policy and the advancement of people's life concepts, the incidence of advanced maternal age has increased day by day [5–7]. At the same time, the comorbidities of elderly women during pregnancy have become more prominent, especially abnormal thyroid function [8, 9]. Among them, thyroid hormone is of great significance in organ metabolism, growth and development. Once thyroid function is impaired, it can directly affect the level of thyroid hormone, threaten maternal metabolism, and cause varying degrees of damage to the growth and development of the fetus. Therefore, it is the key to explore the relationship between thyroid hormones and pregnancy outcomes in advanced women [10, 11]. The results showed that there were significant differences in the serum levels of TSH, FT3, FT4, IgA, IgG, and IgM among the three groups. The incidence of adverse pregnancy outcomes in group C is lower than that in group A and group B. The birth weight and Apgar score of newborns in group A and group B are lower than those in group C. Our results suggest that there are great differences in thyroid hormone and immune ability between elderly parturient women with thyroid diseases and normal elderly parturient women. Therefore, TSH has a great impact on the pregnancy outcomes of elderly parturient women. An abnormal TSH level can increase the risk of adverse pregnancy outcomes. Nevertheless, clinical attention should be paid to actively control TSH levels during pregnancy so as to avoid adverse pregnancy outcomes [12, 13].

It has been reported that abnormal thyroid function is usually expressed in a subclinical form without obvious clinical symptoms. However, pregnancy can promote the transformation of subclinical forms of thyroid dysfunction into clinical manifestations. Moreover, in the second trimester of pregnancy, the fetal development speed is accelerated. Fetal thyroid hormones are usually derived from the mother. Once the thyroid function of pregnant women is abnormal, it can directly cause irreversible damage to fetal nerve function. Fetal thyroid tissue usually begins to develop around 10 weeks of gestation. If the TSH level is abnormal, it may directly limit the normal development of the fetus. At the same time, thyroid hormone levels may also affect maternal immune capacity, which is not conducive to pregnancy outcome [14–18]. Therefore, it is very important to pay attention to the determination of maternal TSH levels, which is helpful to avoid thyroid disease during pregnancy and prevent the phenomenon of fetal intelligence decline.

## 5. Conclusion

It has been reported that when the thyroid hormone of elderly women presents an abnormal expression, it can lead to an increase or decrease of thyroid hormone level. With the prolongation of pregnancy time, the levels of FT3 and FT4 in pregnant women with hyperthyroidism are increased, but the TSH level is decreased significantly. In addition, the abnormal expression levels of TSH, FT3, and FT4 can directly affect the levels of IgA, IgG, and IgM and reduce the immune ability of puerperia. Therefore, for pregnant women with too low or too high TSH levels, we should pay attention to them as soon as possible, choose a reasonable and effective treatment plan for control in a timely manner, and provide effective monitoring to avoid adverse pregnancy outcomes [22–27]. In conclusion, TSH level has a great effect on the pregnancy outcomes of elderly women, which should be paid more attentions in clinical practice. It is of great significance to actively control the TSH level in preventing adverse pregnancy outcomes.

## Figures and Tables

**Table 1:** The comparison results of three groups of thyroid hormone indexes.

Groups	Cases	TSH (*μ*IU/ml)	FT3 (pmol/L)	FT4 (pmol/L)
Group A	20	0.21 ± 0.06	6.51 ± 1.17	23.18 ± 2.14
Group B	35	12.33 ± 3.11	2.24 ± 0.64	2.25 ± 0.65
Group C	42	2.57 ± 0.75	3.67 ± 1.12	3.69 ± 1.13
*F*		340.750	119.560	1981.810
*P*		0.001	0.001	0.001

**Table 2:** The comparison results of three groups of immune indexes.

Groups	Cases	IgA	IgG	IgM
Group A	20	1.85 ± 0.51	10.79 ± 2.58	1.71 ± 0.47
Group B	35	1.33 ± 0.34	9.20 ± 2.06	1.05 ± 0.25
Group C	42	1.64 ± 0.42	9.86 ± 2.18	1.23 ± 0.31
*F*		11.060	3.260	25.780
*P*		0.001	0.043	0.001

**Table 3:** The comparison of adverse pregnancy outcomes among the three groups.

Groups	Cases	Cesarean section	Premature birth	Birth defects	Healthy term infants	Incidence rates
Group A	20	2 (10.00)	1 (5.00)	1 (5.00)	16 (80.00)	4 (20.00)
Group B	35	3 (8.57)	2 (5.71)	1 (2.86)	29 (82.86)	6 (17.14)
Group C	42	1 (2.38)	0 (0.00)	0 (0.00)	41 (97.62)	1 (2.38)
*χ* ^*2*^						6.017
*P*						0.049

**Table 4:** The comparison results of neonatal status of the three groups.

Groups	Cases	Birth weight (g)	Apgar scores
Group A	20	3028.57 ± 123.54	9.22 ± 0.36
Group B	35	3105.66 ± 120.78	9.30 ± 0.44
Group C	42	3352.49 ± 150.69	9.78 ± 0.20
*F*		51.320	27.510
*P*		0.001	0.001

## Data Availability

The simulation experiment data used to support the findings of this study are available from the corresponding author upon request.
